# Stationary Distribution and Extinction of a Stochastic Brucellosis Model with Standard Incidence

**DOI:** 10.1155/2022/4617685

**Published:** 2022-05-29

**Authors:** Dilnaray Iskandar, Xamxinur Abdurahman, Ahmadjan Muhammadhaji

**Affiliations:** College of Mathematics and System Sciences, Xinjiang University, Urumqi 830046, China

## Abstract

In this paper, we proposed a stochastic SVEI brucellosis model with stage structure by introducing the effect of environmental white noise on transmission dynamics of brucellosis. By Has'minskii theory and constructing suitable Lyapunov functions, we established sufficient conditions on the existence of ergodic stationary distribution for the considered model. Moreover, we also established sufficient condition for extinction of the disease. Finally, two examples with numerical simulations are given to illustrate the main results of this paper.

## 1. Introduction

Brucellosis, which is recognized as a major public health problem, is a serious and economically devastating zoonosis which can infect animals, such as sheep, cattle, pig, and dogs. The disease is caused by bacteria of the genus *Brucella*, of which there are six species: *B. abortus*, *B. melitensis*, *B. suis*, *B. ovis*, *B. canis*, and *B. neotomae* [1]. *Brucella* can survive for long periods in dust, dung, water, slurry, aborted fetuses, soil, meat, and dairy products. In animals, brucellosis can be infected by contact with the infected animals (direct way of infection) and by contact of polluted environment (indirect way of transmission), and the disease mainly affects reproduction and fertility and reduces survival of newborns [2]. Brucellosis also can infect human being; the main transmission sources of human brucellosis include exposure to a contaminated environment by infected animals, direct contact with infected animals, and the ingestion of fresh milk or dairy products prepared from unpasteurized milk and unheated meat and animal liver [3]; there is no recorded cases of the infection between humans. Most of the human brucellosis cases are infected by *Brucella melitensis* (which is infected in sheep and goats), accounting for 84.5% of the total cases [4]. In humans, disease-related mortality is negligible, but the illness can last for several years [5]. Therefore, the key to solve the problem of this public health problem is the elimination of animal brucellosis.

It is worth noting that, mathematical models are widely used not only to study the transmission dynamics of brucellosis, but also to study the epidemiological characteristics of brucellosis [1–8]. Recently, the authors in [6] presented a sheep brucellosis model with immigration and proportional birth, considering both direct and indirect transmission. In [7], the authors proposed a multigroup SEIRV dynamical model with bidirectional mixed cross infection between cattle and sheep and investigated the influence of cross infection of mixed feeding on the brucellosis transmission. In [8], the authors proposed the following deterministic brucellosis transmission model:

((1)) $$\begin{array}{c} \left\{\begin{array}{c} \frac{dS_{2}}{dt}=\eta_{1}S_{1}-\beta S_{2}I-\theta S_{2}-\mu_{2}S_{2}+\delta V,\\ \frac{dV}{dt}=\theta S_{2}-\varepsilon \beta VI-\left(\mu_{2}+\delta \right)V,\\ \frac{dE}{dt}=\beta \varepsilon VI+\beta S_{2}I-\left(\mu_{2}+\eta_{2}\right)E,\\ \frac{dI}{dt}=\eta_{2}E-\left(\mu_{2}+c\right)I, \end{array}\right. \end{array}$$

and studied the dynamical behavior of the model, where sheep population is classified into five compartments: the susceptible young sheep *S*_1_(*t*), the susceptible adult (or sexually mature) sheep *S*_2_(*t*), the vaccinated sheep *V*(*t*), the exposed sheep *E*(*t*), and the infectious sheep *I*(*t*). *A* and *b* are the input number of young sheep and the natural birth rate of sheep, and *τ* is the extent of the birth being delayed. *μ*_1_ and *μ*_2_ are the young sheep natural mortality rate and the elimination rate of adult sheep. *η*_1_ and *η*_2_ are the transfer rate from young sheep to adult sheep and exposed sheep to infected sheep. *d* is the output number of young sheep, *δ* is the vaccination rate, *β* is sheep-to-sheep transmission rate, *ε* is the ineffective vaccination rate, and *c* is the elimination rate caused by brucellosis. All the parameters are assumed to be positive.

However, the epidemics in the real world are often disturbed by some uncertain factors, such as environmental white noises. Therefore, it is difficult to describe these epidemic dynamics by using determined differential equation [9]. Thus, the deterministic models has some limitations in mathematical modeling of epidemics, and it is quite difficult to fitting data perfectly and to predicting the future dynamics of the epidemic system. In the past years, there has been a lot of researchers who are interested in the stochastic dynamical models [3, 9–28]. In particular, the stochastic epidemic models have been extensively studied [3, 10–25]. For example, in [3], the authors proposed and studied a periodic stochastic brucellosis model and obtained some conditions on the existence of nontrivial positive periodic solution of the model. In [11], the authors studied a stochastic SIRS epidemic model with standard incidence rate and partial immunity and obtained sufficient conditions on the extinction and existence of a stationary probability measure for the disease of the system. In [12], the authors studied a kind of stochastic SEIR epidemic model with standard incidence and obtained sufficient conditions for the existence of stationary distribution and the extinction of the disease in the system. In [24], the authors discussed a stochastic SIRS epidemic model with logistic growth and nonlinear incidence and obtained sufficient conditions on the ergodic stationary distribution and extinction of the considered model.

On the other hand, there are different approaches used in the literature to introduce random perturbations into population models, both from a mathematical and biological perspective [3, 9–28]. In this paper, in light of the above analysis and reasons, we consider the stochastic perturbations for deterministic system (1) and we employ the approach used in Mao et al. [26] and assume that the parameters involved in the model always fluctuate around some average value due to continuous fluctuations in the environment. This approach is reasonable and well justified biologically [27, 28]. By this approach, we study a stochastic *S*_1_*S*_2_*VEI* brucellosis model with standard incidence, and we assume that the environmental white noise affects the natural mortality rate, the elimination rate, transfer rate, and transmission rate. In order to obtain the stochastic *S*_1_*S*_2_*VEI* brucellosis model, we let *X*(*t*) = (*S*_1_(*t*), *S*_2_(*t*), *V*(*t*), *E*(*t*), *I*(*t*))^*T*^, and then it is appropriate to model *X* = (*S*_1_, *S*_2_, *V*, *E*, *I*)^*T*^ as a Markov process; thus, from [15] and model (1), we can get the following properties when 0 ≤ Δ*t* ≪ 1, the conditional mean

(2) $$\begin{array}{c} E\left[S_{1}\left(t+\Delta t\right)-S_{1}\left(t\right)\;|\;X=x\right]\approx \left[A+\frac{b\left(S_{2}+V\right)}{1+\tau \left(S_{2}+V\right)}-\left(\mu_{1}+d+\eta_{1}\right)S_{1}\right]\Delta t,\\ E\left[S_{2}\left(t+\Delta t\right)-S_{2}\left(t\right)\;|\;X=x\right]\approx \left[\eta_{1}S_{1}-\beta S_{2}I-\theta S_{2}-\mu_{2}S_{2}+\delta V\right]\Delta t,\\ E\left[V\left(t+\Delta t\right)-V\left(t\right)\;|\;X=x\right]\approx \left[\theta S_{2}-\varepsilon \beta VI-\left(\mu_{2}+\delta \right)V\right]\Delta t,\\ E\left[E\left(t+\Delta t\right)-E\left(t\right)\;|\;X=x\right]\approx \left[\beta \varepsilon VI+\beta S_{2}I-\left(\mu_{2}+\eta_{2}\right)E\right]\Delta t,\\ E\left[I\left(t+\Delta t\right)-I\left(t\right)\;|\;X=x\right]\approx \left[\eta_{2}E-\left(\mu_{2}+c\right)I\right]\Delta t, \end{array}$$

and the conditional covariance

(3) $$\begin{array}{c} \text{Var}\left[S_{1}\left(t+\Delta t\right)-S_{1}\left(t\right)\;|\;X=x\right]\approx \sigma_{1}^{2}S_{1}^{2}\Delta t,\\ \text{Var}\left[S_{2}\left(t+\Delta t\right)-S_{2}\left(t\right)\;|\;X=x\right]\approx \sigma_{2}^{2}S_{2}^{2}\Delta t,\\ \text{Var}\left[V\left(t+\Delta t\right)-V\left(t\right)\;|\;X=x\right]\approx \sigma_{3}^{2}V^{2}\Delta t,\\ \text{Var}\left[E\left(t+\Delta t\right)-E\left(t\right)\;|\;X=x\right]\approx \sigma_{4}^{2}E^{2}\Delta t,\\ \text{Var}\left[I\left(t+\Delta t\right)-I\left(t\right)\;|\;X=x\right]\approx \sigma_{5}^{2}I^{2}\Delta t. \end{array}$$

Then, we derive the following stochastic form of system (1)

(4) $$\begin{array}{c} \left\{\begin{array}{c} dS_{1}\left(t\right)=\left[A+\frac{b\left(S_{2}+V\right)}{1+\tau \left(S_{2}+V\right)}-\left(\mu_{1}+d+\eta_{1}\right)S_{1}\right]dt+\sigma_{1}S_{1}dB_{1}\left(t\right),\\ dS_{2}\left(t\right)=\left[\eta_{1}S_{1}-\beta S_{2}I-\theta S_{2}-\mu_{2}S_{2}+\delta V\right]dt+\sigma_{2}S_{2}dB_{2}\left(t\right),\\ dV\left(t\right)=\left[\theta S_{2}-\varepsilon \beta VI-\left(\mu_{2}+\delta \right)V\right]dt+\sigma_{3}VdB_{3}\left(t\right),\\ dE\left(t\right)=\left[\beta \varepsilon VI+\beta S_{2}I-\left(\mu_{2}+\eta_{2}\right)E\right]dt+\sigma_{4}EdB_{4}\left(t\right),\\ dI\left(t\right)=\left[\eta_{2}E-\left(\mu_{2}+c\right)I\right]+\sigma_{5}IdB_{5}\left(t\right), \end{array}\right. \end{array}$$

where *B*_1_(*t*), *B*_2_(*t*), *B*_3_(*t*), *B*_4_(*t*), and *B*_5_(*t*) are the standard one-dimensional independent Brownian motions and *σ*_*i*_^2^ > 0(*i* = 1, 2, 3, 4, 5) are the intensity of the white noises.

The main purpose of the paper is to obtain the conditions for the existence of ergodic stationary distribution and extinction of the disease for model (4).

This paper is organized as follows. In Section 2, we present some preliminaries which will be used in the following analysis. In Section 3, we show that there is a unique global positive solution of system (4). In Section 4, we prove the existence of ergodic stationary distribution for system (4) under certain conditions. In Section 5, we establish sufficient conditions for the disease extinction.

## 2. Preliminaries

Throughout this paper, let (*Ω*, *F*, *ℙ*) be a complete probability space with a filtration {*F*_*t*_}_*t*≥0_ satisfying the usual conditions (i.e., it is increasing and right continuous, while *F*_0_ contains all *ℙ* -null sets); *B*_*i*_(*t*)(*i* = 1, 2, 3, 4) are defined on this complete probability space, and also let ℝ_+_^*d*^ = {*x* ∈ ℝ^*d*^ : *x*_*i*_ > 0, 1 ≤ *i* ≤ *d*}.

In general, consider the *d*-dimensional stochastic differential equation

(5) $$\begin{array}{c} dx\left(t\right)=f\left(x\left(t\right),t\right)dt+g\left(x\left(t\right),t\right)dB\left(t\right)\;\text{for }\left[t_{0},\infty \right], \end{array}$$

with initial value *x*(0) = *x*_0_ ∈ ℝ^*d*^. *B*(*t*) denotes an *n*-dimensional standard Brownian motion defined on the complete probability space (*Ω*, *F*, {*F*_*t*_}_*t*≥0_, *ℙ*). *C*^2,1^(ℝ^*d*^ × [*t*_0_, ∞]; ℝ_+_) denotes the family of all nonnegative functions *V*(*x*, *t*) defined on ℝ^*d*^ × [*t*_0_, ∞] such that they are continuously twice differentiable in *x* and once in *t*. The differential operator *L* of equation (5) is defined by [16].

(6) $$\begin{array}{c} Ł=\frac{\partial }{\partial t}+\overset{d}{\underset{i=1}{\sum }}f_{i}\left(x,t\right)\frac{\partial }{\partial x_{i}}+\frac{1}{2}\overset{d}{\underset{i,j=1}{\sum }}{\left[g^{T}\left(x,t\right)g\left(x,t\right)\right]}_{ij}\frac{\partial^{2}}{\partial x_{i}\partial x_{j}}. \end{array}$$

If *L* acts on a function *V* ∈ *C*^2,1^(ℝ^*d*^ × [*t*_0_, ∞]; ℝ_+_), then

(7) $$\begin{array}{c} LV\left(x,t\right)=V_{t}\left(x,t\right)+V_{x}\left(x,t\right)f\left(x,t\right)+\frac{1}{2}trace\left[g^{T}\left(x,t\right)V_{xx}\left(x,t\right)g\left(x,t\right)\right], \end{array}$$

where *V*_*t*_ = *∂V*/*∂t*, *V*_*x*_ = ((*∂V*/*∂x*_1_), ⋯, (*∂V*/*∂x*_*d*_)), *V*_*xx*_ = (*∂*^2^*V*/*∂x*_*i*_*∂x*_*j*_)_*d*×*d*_. By Itô's formula, if *x*(*t*) ∈ ℝ^*d*^, then

(8) $$\begin{array}{c} dV\left(x\left(t\right),t\right)=LV\left(x\left(t\right),t\right)dt+V_{x}\left(x\left(t\right),t\right)g\left(x\left(t\right),t\right)dB\left(t\right). \end{array}$$

Next, we present a result about the existence of stationary distribution (see Has'minskii [17]).

Let *X*(*t*) be a homogeneous Markov process in *E*_*d*_ (*E*_*d*_ denotes *d*-dimensional Euclidean space) and be described by the following stochastic differential equation:

(9) $$\begin{array}{c} dX\left(t\right)=b\left(X\right)dt+\overset{k}{\underset{r=1}{\sum }}g_{r}\left(X\right)dB_{r}\left(t\right). \end{array}$$

The diffusion matrix is defined as follows:

(10) $$\begin{array}{c} A\left(x\right)=\left(a_{ij}\left(x\right)\right),a_{ij}\left(x\right)=\overset{k}{\underset{r=1}{\sum }}g_{r}^{i}\left(x\right)g_{r}^{j}\left(x\right). \end{array}$$

**Lemma 1 .**

The Markov process *X*(*t*) has a unique ergodic stationary distribution *Π*(·) if there exists a bounded domain *D* ⊂ *E*_*d*_ with regular boundary Γ and

*A*_1_: there is a positive number *M* such that ∑_*i*,*j*=1_^*d*^*a*_*ij*_(*x*)*ξ*_*i*_*ξ*_*j*_ ≥ *M*|*ξ*|^2^, *x* ∈ *D*, *ξ* ∈ ℝ^*d*^.

*A*_2_: there exists a nonnegative *C*^2^-function *V* such that *LV* is negative for any *E*_*d*_\*D*. Then

(11) $$\begin{array}{c} {\mathbb{P}}_{x}\left\{\underset{T⟶\infty }{\lim}\frac{1}{T}\int_{0}^{T}f\left(x\left(t\right)\right)dt=\int_{E_{d}}f\left(x\right)\Pi \left(dx\right)\right\}=1, \end{array}$$

for all *x* ∈ *E*_*d*_, where *f*(·) is a function integrable with respect to the measure *π*.

## 3. Main Results

### 3.1. Existence and Uniqueness of the Positive Solution

In studying the dynamical behavior of an epidemic model, the first importance is whether the solution is global and positive. Hence, in the following theorem, we will study the existence and uniqueness of the global positive solution, which is a prerequisite for researching the long-term behavior of model (4).

**Theorem 1 .**

For any initial value *X*_0_ = (*S*_1_(0), *S*_2_(0), *V*(0), *E*(0), *I*(0)) ∈ ℝ_+_^5^, there is a unique solution *X*(*t*) = (*S*_1_(*t*), *S*_2_(*t*), *V*(*t*), *E*(*t*), *I*(*t*)) of system (4) on *t* ≥ 0, and the solution will remain in ℝ_+_^5^ with probability one.

**Proof**

Since the coefficients of system (4) satisfy the local Lipschitz condition, then for any initial value (*S*_1_(0), *S*_2_(0), *V*(0), *E*(0), *I*(0)) ∈ ℝ_+_^5^, there is a unique local solution (*S*_1_(*t*), *S*_2_(*t*), *V*(*t*), *E*(*t*), *I*(*t*)) on [0, *τ*_*e*_), where *τ*_*e*_ is the explosion time [16]. To show this solution is global, we only need to prove that *τ*_*e*_ = ∞ a.s. To this end, let *n*_0_ > 0 be sufficiently large such that every component of *X*_0_ lying within the interval [(1/*n*_0_), *n*_0_]. For each integer *n* > *n*_0_, define the stopping time as follows:

(12) $$\begin{array}{c} \tau_{n}=\inf\left\{t\in \left[0,\tau_{e}\right)\text{: }\min\left\{S_{1}\left(t\right),S_{2}\left(t\right),V\left(t\right),E\left(t\right),I\left(t\right)\right\}\leq \frac{1}{n}\;\text{or }\max\left\{S_{1}\left(t\right),S_{2}\left(t\right),V\left(t\right),E\left(t\right),I\left(t\right)\right\}\geq n\right\}. \end{array}$$

Throughout this paper, we set inf∅ = ∞ (as usual ∅ denotes the empty set). It is easy to see that *τ*_*n*_ is increasing as *n*⟶∞. Let *τ*_∞_ = lim_*n*⟶∞_*τ*_*n*_, then *τ*_∞_ ≤ *τ*_*e*_ a.s. In what follows, we need to verify *τ*_∞_ = ∞ a.s. If this assertion is violated, there is a constant *T* > 0 and an *ε* ∈ (0, 1) such that *ℙ*{*τ*_∞_ ≤ *T*} > *ε*. As a result, there exists an integer *n*_1_ ≥ *n*_0_ such that

(13) $$\begin{array}{c} \mathbb{P}\left\{\tau_{n}\leq T\right\}\geq \varepsilon ,n\geq n_{1}. \end{array}$$

Define a *C*^2^-function V: ℝ_+_^5^⟶ℝ_+_ by

(14) $$\begin{array}{c} V\left(S_{1},S_{2},V,E,I\right)=\left(S_{1}-1-\ln S_{1}\right)+\left(S_{2}-1-\ln S_{2}\right)+\left(V-1-\ln V\right)+\left(E-1-\ln E\right)+\left(I-1-\ln I\right). \end{array}$$

Using It$\hat{o}$'s formula, we have

(15) $$\begin{array}{c} dV\left(S_{1}S_{2},V,E,I\right)=LV\left(S_{1}S_{2},V,E,I\right)dt+\sigma_{1}\left(S_{1}-1\right)dB_{1}\left(t\right)+\sigma_{2}\left(S_{2}-1\right)dB_{2}\left(t\right)+\sigma_{3}\left(V-1\right)dB_{3}\left(t\right)+\sigma_{4}\left(E-1\right)dB_{4}\left(t\right)+\sigma_{5}\left(I-1\right)dB_{5}\left(t\right), \end{array}$$

where

(16) $$\begin{array}{c} LV=\left(1-\frac{1}{S_{1}}\right)\left(A+\frac{b\left(S_{2}+V\right)}{1+\tau \left(S_{2}+V\right)}-\left(\mu_{1}+d+\eta_{1}\right)S_{1}\right)+\left(1-\frac{1}{S_{2}}\right)\left(\eta_{1}S_{1}-\beta S_{2}I-\theta S_{2}-\mu_{2}S_{2}+\delta V\right)+\left(1-\frac{1}{V}\right)\left(\theta S_{2}-\varepsilon \beta VI-\left(\mu_{2}+\delta \right)V\right)+\left(1-\frac{1}{E}\right)\left(\beta \varepsilon VI+\beta S_{2}I-\left(\mu_{2}+\eta_{2}\right)E\right)+\left(\left(1-\frac{1}{I}\right)\left(\eta_{2}E-\left(\mu_{2}+c\right)I\right)\right.+\frac{\sigma_{1}^{2}+\sigma_{2}^{2}+\sigma_{3}^{2}+\sigma_{4}^{2}+\sigma_{5}^{2}}{2}. \end{array}$$

By applying the following invariant set of model (1) which is obtained in [8]

(17) $$\begin{array}{c} \Omega =\left\{\left(S_{1},S_{2},V,E,I\right)\in R_{+}^{5}:S_{1}+S_{2}+V+E+I\leq \frac{A\tau +b}{\mu \tau }\right\}, \end{array}$$

and from the following inequalities

(18) $$\begin{array}{c} \frac{b\left(S_{2}+V\right)}{1+\tau \left(S_{2}+V\right)}\leq \frac{b}{\tau },I\beta \left(\varepsilon +1\right)\leq \frac{\beta \left(\varepsilon +1\right)\left(A\tau +b\right)}{\mu \tau }, \end{array}$$

and also cancel the items less than zero, so we have

(19) $$\begin{array}{c} LV=A+\frac{b\left(S_{2}+V\right)}{1+\tau \left(S_{2}+V\right)}+\mu_{1}+d+\eta_{1}+\beta I+\theta +4\mu_{2}+\varepsilon \beta I+\delta +\eta_{2}+c-\left(\mu_{1}+d\right)S_{1}-\frac{A}{S_{1}}-\frac{b\left(S_{2}+V\right)}{S_{1}\left[1+\tau \left(S_{2}+V\right)\right]}-\mu_{2}\left(S_{2}+V+E+I\right)-\frac{\eta_{1}S_{1}}{S_{2}}-\frac{\delta V}{S_{2}}-\frac{\theta S_{2}}{V}-\frac{\beta \varepsilon VI}{E}-\frac{\beta S_{2}I}{E}-cI-\frac{\eta_{2}E}{I}+\frac{\sigma_{1}^{2}+\sigma_{2}^{2}+\sigma_{3}^{2}+\sigma_{4}^{2}+\sigma_{5}^{2}}{2}\leq A+\frac{b}{\tau }+\frac{\beta \left(\varepsilon +1\right)\left(A\tau +b\right)}{\mu \tau }+\mu_{1}+d+\eta_{1}+\theta +4\mu_{2}+\delta +\eta_{2}+c+\frac{\sigma_{1}^{2}+\sigma_{2}^{2}+\sigma_{3}^{2}+\sigma_{4}^{2}+\sigma_{5}^{2}}{2}=\zeta . \end{array}$$

Since *ζ* is positive constant which is independent of *S*_1_, *S*_2_, *V*, *E*, *I*, and *t*, we can get

(20) $$\begin{array}{c} dV\left(S_{1}S_{2},V,E,I\right)\leq \zeta dt+\sigma_{1}\left(S_{1}-1\right)dB_{1}\left(t\right)+\sigma_{2}\left(S_{2}-1\right)dB_{2}\left(t\right)+\sigma_{3}\left(V-1\right)dB_{3}\left(t\right)+\sigma_{4}\left(E-1\right)dB_{4}\left(t\right)+\sigma_{5}\left(I-1\right)dB_{5}\left(t\right). \end{array}$$

Integrating both sides (20) from 0 to *T*∧*τ*_*ε*_ and taking expectations, then we can obtain

(21) $$\begin{array}{c} EV\left(S_{1}\left(\tau_{\varepsilon }\wedge T\right),S_{2}\left(\tau_{\varepsilon }\wedge T\right),V\left(\tau_{\varepsilon }\wedge T\right),E\left(\tau_{\varepsilon }\wedge T\right),I\left(\tau_{\varepsilon }\wedge T\right)\right)\leq V\left(S_{1}\left(0\right),S_{2}\left(0\right),V\left(0\right),E\left(0\right),I\left(0\right)\right)+\zeta T<\infty . \end{array}$$

Set *Ω*_*ε*_ = {*τ*_*ε*_ ≤ *t*} for *n* ≥ *n*_1_ by (13), *P*(*Ω*_*n*_) ≥ *ε*. Notice that for every *ω* ∈ *Ω*_*ε*_, there is at least one of *S*_1_(*τ*_*ε*_, *ω*), *S*_2_(*τ*_*ε*_, *ω*), *V*(*τ*_*ε*_, *ω*), *E*(*τ*_*ε*_, *ω*), and *I*(*τ*_*ε*_, *ω*) that equal either *n* or 1/*n*. Hence, *S*_1_(*τ*_*ε*_, *ω*), *S*_2_(*τ*_*ε*_, *ω*), *V*(*τ*_*ε*_, *ω*), *E*(*τ*_*ε*_, *ω*), and *I*(*τ*_*ε*_, *ω*) are no less than

(22) $$\begin{array}{c} n-1-\log n\text{ or }\frac{1}{n}-1-\log n. \end{array}$$

Consequently,

(23) $$\begin{array}{c} \begin{array}{c} V\left(S_{1}\left(\tau_{\varepsilon },\omega \right),S_{2}\left(\tau_{\varepsilon },\omega \right),V\left(\tau_{\varepsilon },\omega \right),E\left(\tau_{\varepsilon },\omega \right),I\left(\tau_{\varepsilon },\omega \right)\right)\geq \left(n-1-\log n\right)\wedge \left(\frac{1}{n}-1-\log n\right), \end{array} \end{array}$$

where *a*∧*b* donates the minimum of *a* and *b*. In view of (21) and (23) we have

(24) $$\begin{array}{c} V\left(S_{1}\left(0\right),S_{2}\left(0\right),V\left(0\right),E\left(0\right),I\left(0\right)\right)+\zeta T\geq E\left[1_{\Omega }\left(\omega \right)V\left(S_{1}\left(\tau_{\varepsilon }\wedge T\right),S_{2}\left(\tau_{\varepsilon }\wedge T\right),V\left(\tau_{\varepsilon }\wedge T\right),E\left(\tau_{\varepsilon }\wedge T\right),I\left(\tau_{\varepsilon }\wedge T\right)\right)\right]\geq \tilde{\delta }\left\{\left(n-1-\log n\right)\wedge \left(\frac{1}{n}-1+\log n\right)\right\}, \end{array}$$

where 1_*Ω*_(*ω*) is the indicator function of *Ω*_*n*_. Let *n*⟶∞ leads to the contradiction

(25) $$\begin{array}{c} \infty >V\left(S_{1}\left(0\right),S_{2}\left(0\right),V\left(0\right),E\left(0\right),I\left(0\right)\right)+\zeta T=\infty . \end{array}$$

Therefore, we must have *τ*_∞_ = ∞ a.s.

### 3.2. Stationary Distribution and Ergodicity

The difference between model (1) and the stochastic model is that the stochastic model does not have the endemic equilibrium. Hence, we cannot study the persistence of the disease by studying the stability of the endemic equilibrium and turn to check out the existence and uniqueness of the stationary distribution for the system (4) which implies the persistence of the disease in some sense. In this section, based on the theory of Has'minskii [17], we verify that there is an ergodic stationary distribution, which reveals the persistence of the disease.

Define a parameter

(26) $$\begin{array}{c} R_{0}^{s}=\frac{\eta_{1}\eta_{2}\beta \varepsilon \theta }{\left(\mu_{1}+d+\eta_{1}+\left(\sigma_{1}^{2}/2\right)\right)\left(\theta +\mu_{2}+\left(\sigma_{2}^{2}/2\right)\right)\left(\mu_{2}+\eta_{2}+\left(\sigma_{4}^{2}/2\right)\right)\left(\mu_{2}+c+\left(\sigma_{5}^{2}/2\right)\right)}. \end{array}$$

**Theorem 2 .**

Assume that *R*_0_^*s*^ > 1, then system (4) has a unique stationary distribution *Π*(·) and it has the ergodic property.

**Proof**

In view of Theorem 2, we have obtained that for any initial value (*S*_1_(0), *S*_2_(0), *V*(0), *E*(0), *I*(0)) ∈ ℝ_+_^5^), there is a unique global solution (*S*_1_, *S*_2_, *V*, *E*, *I*) ∈ ℝ_+_^5.^.

The diffusion matrix of system (4) is given by

(27) $$\begin{array}{c} A=\left(\begin{array}{ccccc} \sigma_{1}^{2}S_{1}^{2} & 0 & 0 & 0 & 0\\ 0 & \sigma_{2}^{2}S_{2}^{2} & 0 & 0 & 0\\ 0 & 0 & \sigma_{3}^{2}V^{2} & 0 & 0\\ 0 & 0 & 0 & \sigma_{4}^{2}E^{2} & 0\\ 0 & 0 & 0 & 0 & \sigma_{5}^{2}I^{2} \end{array}\right). \end{array}$$

Choose $M=\min_{\left(S_{1},S_{2},V,E,I\right)\in {\bar{D}}_{\sigma }\subset R_{+}^{5}}\left\{\sigma_{1}^{2}S_{1}^{2},\sigma_{1}^{2}S_{2}^{2},\sigma_{3}^{2}V^{2},\sigma_{4}^{2}E^{2},\sigma_{5}^{2}I^{2}\right\}$; one can get that

(28) $$\begin{array}{c} \overset{5}{\underset{i,j=1}{\sum }}a_{ij}\left(S_{1},S_{2},V,E,I\right)\xi_{i}\xi_{j}=\sigma_{1}^{2}S_{1}^{2}\xi_{1}^{2}+\sigma_{1}^{2}S_{2}^{2}\xi_{2}^{2}+\sigma_{3}^{2}V^{2}\xi_{3}^{2}+\sigma_{4}^{2}E^{2}\xi_{4}^{2}+\sigma_{5}^{2}I^{2}\xi_{5}^{2}\geq M{\left|\xi \right|}^{2},\\ \left(S_{1},S_{2},V,E,I\right)\in {\bar{D}}_{\sigma },\xi =\left(\xi_{1},\xi_{2},\xi_{3},\xi_{4},\xi_{5}\right)\in {\mathbb{R}}_{+}^{5}. \end{array}$$

Then the condition *A*_1_ in Lemma 1 is satisfied.

Construct a *C*^2^-function *Q* : ℝ_+_^5^⟶ℝ in the following from

(29) $$\begin{array}{c} Q\left(S_{1},S_{2},V,E,I\right)=M\left(S_{1}+S_{2}+V+E+I-c_{1}\ln S_{1}-c_{2}\ln S_{2}-c_{3}\ln E-c_{4}\ln I-\ln V\right)+\frac{1}{\chi +1}{\left(S_{1}+S_{2}+V+E+I\right)}^{\chi +1}-\ln S_{1}-\ln S_{2}-\ln E-\ln V+\left(S_{1}+S_{2}+V+E+I\right)=MV_{1}+V_{2}+V_{3}+V_{4}+V_{5}+V_{6}, \end{array}$$

where *χ* is a constant satisfying 0 < *χ* < 2*μ*/*σ*_1_^2^∨*σ*_2_^2^∨*σ*_3_^2^∨*σ*_4_^2^∨*σ*_5_^2^,

(30) $$\begin{array}{c} c_{1}=\frac{A}{\mu_{1}+d+\eta_{1}+\left(\sigma_{1}^{2}/2\right)},c_{2}=\frac{A}{\theta +\mu_{2}+\left(\sigma_{2}^{2}/2\right)},c_{3}=\frac{A}{\mu_{2}+\eta_{2}+\left(\sigma_{4}^{2}/2\right)},c_{4}=\frac{A}{\mu_{2}+c+\left(\sigma_{5}^{2}/2\right)}, \end{array}$$

and *M* > 0 satisfies the following condition

(31) $$\begin{array}{c} -M\lambda +C\leq -2, \end{array}$$

where

(32) $$\begin{array}{c} \lambda =5A\left\{{\left[\frac{\eta_{1}\eta_{2}\beta \varepsilon \theta }{\left(\mu_{1}+d+\eta_{1}+\left(\sigma_{1}^{2}/2\right)\right)\left(\theta +\mu_{2}+\left(\sigma_{2}^{2}/2\right)\right)\left(\mu_{2}+\eta_{2}+\left(\sigma_{4}^{2}/2\right)\right)\left(\mu_{2}+c+\left(\sigma_{5}^{2}/2\right)\right)}\right]}^{1/5}-1\right\}=5A\left[{\left(R_{0}^{s}\right)}^{1/5}-1\right]>0, \end{array}$$

(33) $$\begin{array}{c} \begin{array}{c} C=\underset{\left(S_{1},S_{2},V,E,I\right)\varepsilon {\mathbb{R}}_{+}^{5}}{\sup}\left\{-\frac{1}{2}\left[\mu -\frac{1}{2}\sigma \left(\sigma_{1}^{2}\vee \sigma_{2}^{2}\vee \sigma_{3}^{2}\vee \sigma_{4}^{2}\vee \sigma_{5}^{2}\right)\right]\right.\\ \cdot \left(S_{1}^{\chi +1}+S_{2}^{\chi +1}+V^{\chi +1}+E^{\chi +1}+I^{\chi +1}\right)+\mu_{1}+d+\eta_{1}+\theta +3\mu_{2}+\eta_{2}\\ \left.+\delta +A+\frac{b}{\tau }+M\left(\frac{\sigma_{3}^{2}}{2}+\mu_{2}+\delta +\frac{b}{\tau }\right)+\frac{\sigma_{1}^{2}+\sigma_{2}^{2}+\sigma_{3}^{2}+\sigma_{4}^{2}}{2}\right\}. \end{array} \end{array}$$

It is easy to check that

(34) $$\begin{array}{c} \lim\underset{k⟶\infty ,\left(S_{1},S_{2},V,E,I\right)\in {\mathbb{R}}_{+}^{5}\backslash U_{k}}{\inf}Q\left(S_{1},S_{2},V,E,I\right)=\infty , \end{array}$$

where *U*_*k*_ = ((1/*k*), *k*) × ((1/*k*), *k*) × ((1/*k*), *k*) × ((1/*k*), *k*) × ((1/*k*), *k*). Furthermore, *Q*(*S*_1_, *S*_2_, *V*, *E*, *I*) is a continuous function. Hence, *Q*(*S*_1_, *S*_2_, *V*, *E*, *I*) must have a minimum point $\left({\bar{S}}_{1}\left(0\right),{\bar{S}}_{2}\left(0\right),\bar{V}\left(0\right),\bar{E}\left(0\right),\bar{I}\left(0\right)\right)$ in the interior of ℝ_+_^5^. Then we define a nonnegative *C*^2^-function *V* : ℝ_+_^5^⟶ℝ_+_ as follows:

(35) $$\begin{array}{c} V\left(S_{1},S_{2},V,E,I\right)=Q\left(S_{1},S_{2},V,E,I\right)-Q\left({\bar{S}}_{1}\left(0\right),{\bar{S}}_{2}\left(0\right),\bar{V}\left(0\right),\bar{E}\left(0\right),\bar{I}\left(0\right)\right). \end{array}$$

Making use of It$\hat{o}$'s formula, we have

(36) $$\begin{array}{c} LV_{1}=-\left(\mu_{2}\left(S_{2}+V+E+I\right)+\left(\mu_{1}+d\right)S_{1}+\frac{c_{1}A}{S_{1}}+\frac{c_{1}b\left(S_{2}+V\right)}{S_{1}\left[1+\tau \left(S_{2}+V\right)\right]}+\frac{c_{2}\eta_{1}S_{1}}{S_{2}}+\frac{c_{2}\delta V}{S_{2}}+\frac{c_{3}\beta \varepsilon VI}{E}+\frac{c_{3}\beta S_{2}I}{E}+\frac{c_{4}\eta_{2}E}{I}+\frac{\theta S_{2}}{V}\right)-cI+A+\frac{b\left(S_{2}+V\right)}{1+\tau \left(S_{2}+V\right)}+\varepsilon \beta I+c_{2}\beta I+\mu_{2}+\delta +\frac{\sigma_{3}^{2}}{2}+c_{1}\left(\mu_{1}+d+\eta_{1}+\frac{\sigma_{1}^{2}}{2}\right)+c_{2}\left(\theta +\mu_{2}+\frac{\sigma_{2}^{2}}{2}\right)+c_{3}\left(\mu_{2}+\eta_{2}+\frac{\sigma_{4}^{2}}{2}\right)+c_{4}\left(\mu_{2}+c+\frac{\sigma_{5}^{2}}{2}\right). \end{array}$$

Using the inequality $a+b+c+d+e\geq 5\sqrt[{5}]{abcde},a,b,c,d,e>0$ leads to

(37) $$\begin{array}{c} LV_{1}\leq -\left(\frac{c_{1}A}{S_{1}}+\frac{c_{2}\eta_{1}S_{1}}{S_{2}}+\frac{c_{3}\beta \varepsilon VI}{E}+\frac{c_{4}\eta_{2}E}{I}+\frac{\theta S_{2}}{V}\right)+A+\frac{b}{\tau }+\varepsilon \beta I+c_{2}\beta I+\mu_{2}+\delta +\frac{\sigma_{3}^{2}}{2}+c_{1}\left(\mu_{1}+d+\eta_{1}+\frac{\sigma_{1}^{2}}{2}\right)+c_{2}\left(\theta +\mu_{2}+\frac{\sigma_{2}^{2}}{2}\right)+c_{3}\left(\mu_{2}+\eta_{2}+\frac{\sigma_{4}^{2}}{2}\right)+c_{4}\left(\mu_{2}+c+\frac{\sigma_{5}^{2}}{2}\right)\leq -5{\left(c_{1}c_{2}c_{3}c_{4}A\eta_{1}\beta \varepsilon \eta_{2}\theta \right)}^{1/5}+A+\frac{b}{\tau }+\varepsilon \beta I+c_{2}\beta I+\mu_{2}+\delta +\frac{\sigma_{3}^{2}}{2}+c_{1}\left(\mu_{1}+d+\eta_{1}+\frac{\sigma_{1}^{2}}{2}\right)+c_{2}\left(\theta +\mu_{2}+\frac{\sigma_{2}^{2}}{2}\right)+c_{3}\left(\mu_{2}+\eta_{2}+\frac{\sigma_{4}^{2}}{2}\right)+c_{4}\left(\mu_{2}+c+\frac{\sigma_{5}^{2}}{2}\right)=-5{\left(\frac{A^{5}\eta_{1}\beta \varepsilon \eta_{2}\theta }{\left(\mu_{1}+d+\eta_{1}+\left(\sigma_{1}^{2}/2\right)\right)\left(\theta +\mu_{2}+\left(\sigma_{2}^{2}/2\right)\right)\left(\mu_{2}+\eta_{2}+\left(\sigma_{4}^{2}/2\right)\right)\left(\mu_{2}+c+\left(\sigma_{5}^{2}/2\right)\right)}\right)}^{1/5}+5A+\mu_{2}+\delta +\frac{b}{\tau }+\beta I\left(c_{2}+\varepsilon \right)+\frac{\sigma_{3}^{2}}{2}=-5A\left\{{\left[\frac{\eta_{1}\beta \varepsilon \eta_{2}\theta }{\left(\mu_{1}+d+\eta_{1}+\left(\sigma_{1}^{2}/2\right)\right)\left(\theta +\mu_{2}+\left(\sigma_{2}^{2}/2\right)\right)\left(\mu_{2}+\eta_{2}+\left(\sigma_{4}^{2}/2\right)\right)\left(\mu_{2}+c+\left(\sigma_{5}^{2}/2\right)\right)}\right]}^{1/5}-1\right\}+\mu_{2}+\delta +\frac{b}{\tau }+\beta I\left(c_{2}+\varepsilon \right)+\frac{\sigma_{3}^{2}}{2}=-\lambda +\mu_{2}+\delta +\frac{b}{\tau }+\beta I\left(c_{2}+\varepsilon \right)+\frac{\sigma_{3}^{2}}{2}, \end{array}$$

where *λ* is defined in (32).

Similarly

(38) $$\begin{array}{c} LV_{2}={\left(S_{1}+S_{2}+V+E+I\right)}^{\chi }\left[A+\frac{b\left(S_{2}+V\right)}{1+\tau \left(S_{2}+V\right)}-\left(\mu_{1}+d\right)S_{1}-\mu_{2}\left(S_{2}+V+E+I\right)-cI\right]+\frac{1}{2}\chi {\left(S_{1}+S_{2}+V+E+I\right)}^{\chi -1}\times \left(\sigma_{1}^{2}S_{1}^{2}+\sigma_{2}^{2}S_{2}^{2}+\sigma_{3}^{2}V^{2}+\sigma_{4}^{2}E^{+}\sigma_{5}^{2}I^{2}\right)\leq {\left(S_{1}+S_{2}+V+E+I\right)}^{\chi }\left[A+\frac{b}{\tau }-\mu \left(S_{1}+S_{2}+V+E+I\right)\right]+\frac{1}{2}\chi {\left(S_{1}+S_{2}+V+E+I\right)}^{\chi +1}\left(\sigma_{1}^{2}\vee \sigma_{2}^{2}\vee \sigma_{3}^{2}\vee \sigma_{4}^{2}\vee \sigma_{5}^{2}\right)=\left(A+\frac{b}{\tau }\right){\left(S_{1}+S_{2}+V+E+I\right)}^{\chi }-\left[\mu -\frac{1}{2}\chi \left(\sigma_{1}^{2}\vee \sigma_{2}^{2}\vee \sigma_{3}^{2}\vee \sigma_{4}^{2}\vee \sigma_{5}^{2}\right)\right]{\left(S_{1}+S_{2}+V+E+I\right)}^{\chi +1}. \end{array}$$

Then

(39) $$\begin{array}{c} LV_{2}\leq B-\frac{1}{2}\left[\mu -\frac{1}{2}\chi \left(\sigma_{1}^{2}\vee \sigma_{2}^{2}\vee \sigma_{3}^{2}\vee \sigma_{4}^{2}\vee \sigma_{5}^{2}\right)\right]{\left(S_{1}+S_{2}+V+E+I\right)}^{\chi +1}\leq B-\frac{1}{2}\left[\mu -\frac{1}{2}\chi \left(\sigma_{1}^{2}\vee \sigma_{2}^{2}\vee \sigma_{3}^{2}\vee \sigma_{4}^{2}\vee \sigma_{5}^{2}\right)\right]\left(S_{1}^{\chi +1}+S_{2}^{\chi +1}+V^{\chi +1}+E^{\chi +1}+I^{\chi +1}\right), \end{array}$$

where

(40) $$\begin{array}{c} B=\underset{\left(S_{1},S_{2},V,E,I\right)\in {\mathbb{R}}_{+}^{5}}{\sup}\left\{\left(A+\frac{b}{\tau }\right){\left(S_{1}+S_{2}+V+E+I\right)}^{\chi }-\frac{1}{2}\left[\mu -\frac{1}{2}\chi \left(\sigma_{1}^{2}\vee \sigma_{2}^{2}\vee \sigma_{3}^{2}\vee \sigma_{4}^{2}\vee \sigma_{5}^{2}\right)\right]{\left(S_{1}+S_{2}+V+E+I\right)}^{\chi +1}\right\}<\infty . \end{array}$$

We can also get

(41) $$\begin{array}{c} \begin{array}{c} LV_{3}=-\frac{A}{S_{1}}-\frac{b\left(S_{2}+V\right)}{S_{1}\left[1+\tau \left(S_{2}+V\right)\right]}+\left(\mu_{1}+d+\eta_{1}\right)+\frac{\sigma_{1}^{2}}{2}, \end{array} \end{array}$$

(42) $$\begin{array}{c} \begin{array}{c} LV_{4}=-\frac{\eta_{1}S_{1}}{S_{2}}+\beta I+\theta +\mu_{2}-\frac{\delta V}{S_{2}}+\frac{\sigma_{2}^{2}}{2}, \end{array} \end{array}$$

(43) $$\begin{array}{c} \begin{array}{c} LV_{5}=-\frac{\beta \varepsilon VI}{E}-\frac{\beta S_{2}I}{E}+\left(\mu_{2}+\eta_{2}\right)+\frac{\sigma_{4}^{2}}{2}, \end{array} \end{array}$$

(44) $$\begin{array}{c} \begin{array}{c} LV_{6}=-\frac{\theta S_{2}}{V}+\varepsilon \beta I+\left(\mu_{2}+\delta \right)+\frac{\sigma_{3}^{2}}{2}, \end{array} \end{array}$$

(45) $$\begin{array}{c} LV_{7}=A+\frac{\left(S_{2}+V\right)}{1+\tau \left(S_{2}+V\right)}-\left(\mu_{1}+d\right)S_{1}-\mu_{2}\left(S_{2}+V+E+I\right)-cI\leq A+\frac{b}{\tau }-\left(\mu_{1}+d\right)S_{1}-\mu_{2}\left(S_{2}+V+E+I\right). \end{array}$$

Hence, by (37)-(45), we obtain

(46) $$\begin{array}{c} LV\leq -M\lambda +M\beta I\left(c_{2}+\varepsilon +\frac{1+\varepsilon }{M}\right)+B-\frac{1}{2}\left[\mu -\frac{1}{2}\chi \left(\sigma_{1}^{2}\vee \sigma_{2}^{2}\vee \sigma_{3}^{2}\vee \sigma_{4}^{2}\vee \sigma_{5}^{2}\right)\right]\times \left(S_{1}^{\chi +1}+S_{2}^{\chi +1}+V^{\chi +1}+E^{\chi +1}+I^{\chi +1}\right)-\frac{A}{S_{1}}-\frac{b\left(S_{2}+V\right)}{S_{1}\left[1+\tau \left(S_{2}+V\right)\right]}-\frac{\eta_{1}S_{1}}{S_{2}}-\frac{\delta V}{S_{2}}-\frac{\beta \varepsilon VI}{E}-\frac{\beta S_{2}I}{E}-\frac{\theta S_{2}}{V}-\left(\mu_{1}+d\right)S_{1}-\mu_{2}\left(S_{2}+V+E+I\right)+\mu_{1}+d+\eta_{1}+\theta +3\mu_{2}+\eta_{2}+\delta +A+\frac{b}{\tau }+M\left(\frac{\sigma_{3}^{2}}{2}+\mu_{2}+\delta +\frac{b}{\tau }\right)+\frac{\sigma_{1}^{2}+\sigma_{2}^{2}+\sigma_{3}^{2}+\sigma_{4}^{2}}{2}. \end{array}$$

Thus, we can construct a compact subset *D* such that the condition *A*_2_ in Lemma 1 holds. Define the bounded closed set

(47) $$\begin{array}{c} D=\left\{\varepsilon_{1}\leq S_{1}\leq \frac{1}{\varepsilon_{1}},\varepsilon_{2}\leq S_{2}\leq \frac{1}{\varepsilon_{2}},\varepsilon_{3}\leq I\leq \frac{1}{\varepsilon_{3}},\varepsilon_{4}\leq E\leq \frac{1}{\varepsilon_{4}},\varepsilon_{5}\leq V\leq \frac{1}{\varepsilon_{5}}\right\}, \end{array}$$

where *ε*_*i*_ > 0(*i* = 1, 2, 3, 4, 5) are sufficiently small constants satisfying the following conditions:

(48) $$\begin{array}{c} \begin{array}{c} -\frac{1}{\varepsilon_{1}}+F\leq -1, \end{array} \end{array}$$

(49) $$\begin{array}{c} \begin{array}{c} -M\lambda -\frac{\varepsilon_{5}}{\varepsilon_{2}}+C\leq -1, \end{array} \end{array}$$

(50) $$\begin{array}{c} -M\lambda +M\beta \varepsilon_{3}\left(\frac{1+\varepsilon }{M}+c_{2}+\varepsilon \right)+C\leq -1, \end{array}$$

(51) $$\begin{array}{c} -\frac{\beta \varepsilon_{2}\varepsilon_{3}}{\varepsilon_{4}}+F\leq -1, \end{array}$$

(52) $$\begin{array}{c} -\frac{\theta S_{2}}{\varepsilon_{5}}+F\leq -1, \end{array}$$

(53) $$\begin{array}{c} -\frac{1}{4}\left[\mu -\frac{1}{2}\chi \left(\sigma_{1}^{2}\vee \sigma_{2}^{2}\vee \sigma_{3}^{2}\vee \sigma_{4}^{2}\vee \sigma_{5}^{2}\right)\right]\frac{1}{\varepsilon_{1}^{\chi +1}}+G\leq -1, \end{array}$$

(54) $$\begin{array}{c} -\frac{1}{4}\left[\mu -\frac{1}{2}\chi \left(\sigma_{1}^{2}\vee \sigma_{2}^{2}\vee \sigma_{3}^{2}\vee \sigma_{4}^{2}\vee \sigma_{5}^{2}\right)\right]\frac{1}{\varepsilon_{2}^{\chi +1}}+H\leq -1, \end{array}$$

(55) $$\begin{array}{c} -\frac{1}{4}\left[\mu -\frac{1}{2}\chi \left(\sigma_{1}^{2}\vee \sigma_{2}^{2}\vee \sigma_{3}^{2}\vee \sigma_{4}^{2}\vee \sigma_{5}^{2}\right)\right]\frac{1}{\varepsilon_{4}^{\chi +1}}+J\leq -1, \end{array}$$

(56) $$\begin{array}{c} -\frac{1}{4}\left[\mu -\frac{1}{2}\chi \left(\sigma_{1}^{2}\vee \sigma_{2}^{2}\vee \sigma_{3}^{2}\vee \sigma_{4}^{2}\vee \sigma_{5}^{2}\right)\right]\frac{1}{\varepsilon_{3}^{\chi +1}}+K\leq -1, \end{array}$$

(57) $$\begin{array}{c} -\frac{1}{4}\left[\mu -\frac{1}{2}\chi \left(\sigma_{1}^{2}\vee \sigma_{2}^{2}\vee \sigma_{3}^{2}\vee \sigma_{4}^{2}\vee \sigma_{5}^{2}\right)\right]\frac{1}{\varepsilon_{5}^{\chi +1}}+L\leq -1, \end{array}$$

where *F*, *G*, *H*, *J*, *K*, and *L* are positive constants which can be seen from (60), (68), (70), (72), (74), and (76), respectively. Note that for sufficiently small *ε*_*i*_, *i* = 1, 2, 3, 4, 5. For convenience, we divide ℝ_+_^5^\*D* into ten domains

(58) $$\begin{array}{c} \begin{array}{c} D_{1}=\left\{\left(S_{1},S_{2},V,E,I\right)\in {\mathbb{R}}_{+}^{5}:0<S_{1}<\varepsilon_{1}\right\},\\ D_{2}=\left\{\left(S_{1},S_{2},V,E,I\right)\in {\mathbb{R}}_{+}^{5}:0<S_{2}<\varepsilon_{2},V\geq \varepsilon_{5}\right\},\\ D_{3}=\left\{\left(S_{1},S_{2},V,E,I\right)\in {\mathbb{R}}_{+}^{5}:0<I<\varepsilon_{3}\right\},\\ D_{4}=\left\{\left(S_{1},S_{2},V,E,I\right)\in {\mathbb{R}}_{+}^{5}:S_{2}\geq \varepsilon_{2},I\geq \varepsilon_{3},0<E<\varepsilon_{4}\right\},\\ D_{5}=\left\{\left(S_{1},S_{2},V,E,I\right)\in {\mathbb{R}}_{+}^{5}:0<V<\varepsilon_{5}S_{2}\geq \varepsilon_{2}\right\},\\ D_{6}=\left\{\left(S_{1},S_{2},V,E,I\right)\in {\mathbb{R}}_{+}^{5}:S_{1}>\frac{1}{\varepsilon_{1}}\right\},\\ D_{7}=\left\{\left(S_{1},S_{2},V,E,I\right)\in {\mathbb{R}}_{+}^{5}:S_{2}>\frac{1}{\varepsilon_{2}}\right\},\\ D_{8}=\left\{\left(S_{1},S_{2},V,E,I\right)\in {\mathbb{R}}_{+}^{5}:I>\frac{1}{\varepsilon_{3}}\right\},\\ D_{9}=\left\{\left(S_{1},S_{2},V,E,I\right)\in {\mathbb{R}}_{+}^{5}:E>\frac{1}{\varepsilon_{4}}\right\},\\ D_{10}=\left\{\left(S_{1},S_{2},V,E,I\right)\in {\mathbb{R}}_{+}^{5}:V>\frac{1}{\varepsilon_{5}}\right\}. \end{array} \end{array}$$

Next, we will show that *LV*(*S*_1_, *S*_2_, *V*, *E*, *I*) ≤ −1 on ℝ_+_^5^\*D*, which is equivalent to proving it on the above ten domains.

**Case 1 .**

If (*S*_1_, *S*_2_, *V*, *E*, *I*) ∈ *D*_1_, one can get that

(59) $$\begin{array}{c} LV\leq -\frac{A}{S_{1}}+M\beta I\left(c_{2}+\varepsilon +\frac{1+\varepsilon }{M}\right)-\frac{1}{2}\left[\mu -\frac{1}{2}\chi \left(\sigma_{1}^{2}\vee \sigma_{2}^{2}\vee \sigma_{3}^{2}\vee \sigma_{4}^{2}\vee \sigma_{5}^{2}\right)\right]\left(S_{1}^{\chi +1}+S_{2}^{\chi +1}+V^{\chi +1}+E^{\chi +1}+I^{\chi +1}\right)+\mu_{1}+d+\eta_{1}+\theta +3\mu_{2}+\eta_{2}+\delta +A+\frac{b}{\tau }+M\left(\frac{\sigma_{3}^{2}}{2}+\mu_{2}+\delta +\frac{b}{\tau }\right)+\frac{\sigma_{1}^{2}+\sigma_{2}^{2}+\sigma_{3}^{2}+\sigma_{4}^{2}}{2}\leq -\frac{A}{S_{1}}+F\leq -\frac{A}{\varepsilon_{1}}+F\leq -1, \end{array}$$

where

(60) $$\begin{array}{c} F=\underset{\left(S_{1},S_{2},V,E,I\right)\in {\mathbb{R}}_{+}^{5}}{\sup}\left\{M\beta I\left(c_{2}+\varepsilon +\frac{1+\varepsilon }{M}\right)-\frac{1}{2}\left[\mu -\frac{1}{2}\chi \left(\sigma_{1}^{2}\vee \sigma_{2}^{2}\vee \sigma_{3}^{2}\vee \sigma_{4}^{2}\vee \sigma_{5}^{2}\right)\right]\times \left(S_{1}^{\chi +1}+S_{2}^{\chi +1}+V^{\chi +1}+E^{\chi +1}+I^{\chi +1}\right)+\mu_{1}+d+\eta_{1}+\theta +3\mu_{2}+\eta_{2}+\delta +A+\frac{b}{\tau }+M\left(\frac{\sigma_{3}^{2}}{2}+\mu_{2}+\delta +\frac{b}{\tau }\right)+\frac{\sigma_{1}^{2}+\sigma_{2}^{2}+\sigma_{3}^{2}+\sigma_{4}^{2}}{2}\right\}. \end{array}$$

According to (48), we have

(61) $$\begin{array}{c} LV\leq -1,\text{for any }\left(S_{1},S_{2},V,E,I\right)\in D_{1}. \end{array}$$

**Case 2 .**

If (*S*_1_, *S*_2_, *V*, *E*, *I*) ∈ *D*_2_, we have

(62) $$\begin{array}{c} LV\leq -M\lambda -\frac{\delta V}{S_{2}}-\frac{1}{2}\left[\mu -\frac{1}{2}\chi \left(\sigma_{1}^{2}\vee \sigma_{2}^{2}\vee \sigma_{3}^{2}\vee \sigma_{4}^{2}\vee \sigma_{5}^{2}\right)\right]\left(S_{1}^{\chi +1}+S_{2}^{\chi +1}+V^{\chi +1}+E^{\chi +1}+I^{\chi +1}\right)+\mu_{1}+d+\eta_{1}+\theta +3\mu_{2}+\eta_{2}+\delta +A+\frac{b}{\tau }+M\left(\frac{\sigma_{3}^{2}}{2}+\mu_{2}+\delta +\frac{b}{\tau }\right)+\frac{\sigma_{1}^{2}+\sigma_{2}^{2}+\sigma_{3}^{2}+\sigma_{4}^{2}}{2}\leq -M\lambda -\frac{\delta V}{S_{2}}+C\leq -M\lambda -\frac{\varepsilon_{5}}{\varepsilon_{2}}+C, \end{array}$$

where *C* is defined in (33).

In view of (49), we can obtain that for sufficiently small *ε*_*i*_(*i* = 2, 5), *LV* ≤ −1 for any (*S*_1_, *S*_2_, *V*, *E*, *I*) ∈ *D*_2_.

**Case 3 .**

If (*S*_1_, *S*_2_, *V*, *E*, *I*) ∈ *D*_3_, one can see that

(63) $$\begin{array}{c} LV\leq -M\lambda +M\beta I\left(c_{2}+\varepsilon +\frac{1+\varepsilon }{M}\right)-\frac{1}{2}\left[\mu -\frac{1}{2}\chi \left(\sigma_{1}^{2}\vee \sigma_{2}^{2}\vee \sigma_{3}^{2}\vee \sigma_{4}^{2}\vee \sigma_{5}^{2}\right)\right]\left(S_{1}^{\chi +1}+S_{2}^{\chi +1}+V^{\chi +1}+E^{\chi +1}+I^{\chi +1}\right)+\mu_{1}+d+\eta_{1}+\theta +3\mu_{2}+\eta_{2}+\delta +A+\frac{b}{\tau }+M\left(\frac{\sigma_{3}^{2}}{2}+\mu_{2}+\delta +\frac{b}{\tau }\right)+\frac{\sigma_{1}^{2}+\sigma_{2}^{2}+\sigma_{3}^{2}+\sigma_{4}^{2}}{2}. \end{array}$$

We obtain that

(64) $$\begin{array}{c} LV\leq -1\text{ for any }\left(S_{1},S_{2},V,E,I\right)\in D_{3}. \end{array}$$

**Case 4 .**

If (*S*_1_, *S*_2_, *V*, *E*, *I*) ∈ *D*_4_, one can see that

(65) $$\begin{array}{c} LV\leq -\frac{\beta S_{2}I}{E}+M\beta I\left(c_{2}+\varepsilon +\frac{1+\varepsilon }{M}\right)-\frac{1}{2}\left[\mu -\frac{1}{2}\chi \left(\sigma_{1}^{2}\vee \sigma_{2}^{2}\vee \sigma_{3}^{2}\vee \sigma_{4}^{2}\vee \sigma_{5}^{2}\right)\right]\left(S_{1}^{\chi +1}+S_{2}^{\chi +1}+V^{\chi +1}+E^{\chi +1}+I^{\chi +1}\right)+\mu_{1}+d+\eta_{1}+\theta +3\mu_{2}+\eta_{2}+\delta +A+\frac{b}{\tau }+M\left(\frac{\sigma_{3}^{2}}{2}+\mu_{2}+\delta +\frac{b}{\tau }\right)+\frac{\sigma_{1}^{2}+\sigma_{2}^{2}+\sigma_{3}^{2}+\sigma_{4}^{2}}{2}\leq -\frac{\beta S_{2}I}{E}+F\leq -\frac{\beta \varepsilon_{2}\varepsilon_{3}}{\varepsilon_{4}}+F. \end{array}$$

In view of (51), we can obtain that for sufficiently small *ε*_*i*_(*i* = 3, 4), *LV* ≤ −1 for any (*S*_1_, *S*_2_, *V*, *E*, *I*) ∈ *D*_4_.

**Case 5 .**

If (*S*_1_, *S*_2_, *V*, *E*, *I*) ∈ *D*_5_, one can see that

(66) $$\begin{array}{c} LV\leq -\frac{\theta S_{2}}{V}+M\beta I\left(c_{2}+\varepsilon +\frac{1+\varepsilon }{M}\right)-\frac{1}{2}\left[\mu -\frac{1}{2}\chi \left(\sigma_{1}^{2}\vee \sigma_{2}^{2}\vee \sigma_{3}^{2}\vee \sigma_{4}^{2}\vee \sigma_{5}^{2}\right)\right]\left(S_{1}^{\chi +1}+S_{2}^{\chi +1}+V^{\chi +1}+E^{\chi +1}+I^{\chi +1}\right)+\mu_{1}+d+\eta_{1}+\theta +3\mu_{2}+\eta_{2}+\delta +A+\frac{b}{\tau }+M\left(\frac{\sigma_{3}^{2}}{2}+\mu_{2}+\delta +\frac{b}{\tau }\right)+\frac{\sigma_{1}^{2}+\sigma_{2}^{2}+\sigma_{3}^{2}+\sigma_{4}^{2}}{2}\leq -\frac{\theta S_{2}}{V}+F\leq -\frac{\theta \varepsilon_{2}}{\varepsilon_{5}}+F. \end{array}$$

We can obtain that for sufficiently small *ε*_*i*_(*i* = 2, 5), *LV* ≤ −1 for any (*S*_1_, *S*_2_, *V*, *E*, *I*) ∈ *D*_5_.

**Case 6 .**

If (*S*_1_, *S*_2_, *V*, *E*, *I*) ∈ *D*_6_, one can see that

(67) $$\begin{array}{c} LV\leq -\frac{1}{4}\left[\mu -\frac{1}{2}\chi \left(\sigma_{1}^{2}\vee \sigma_{2}^{2}\vee \sigma_{3}^{2}\vee \sigma_{4}^{2}\vee \sigma_{5}^{2}\right)\right]S_{1}^{\chi +1}-\frac{1}{4}\left[\mu -\frac{1}{2}\chi \left(\sigma_{1}^{2}\vee \sigma_{2}^{2}\vee \sigma_{3}^{2}\vee \sigma_{4}^{2}\vee \sigma_{5}^{2}\right)\right]\times S_{1}^{\chi +1}-\frac{1}{2}\left[\mu -\frac{1}{2}\chi \left(\sigma_{1}^{2}\vee \sigma_{2}^{2}\vee \sigma_{3}^{2}\vee \sigma_{4}^{2}\vee \sigma_{5}^{2}\right)\right]\left(S_{2}^{\chi +1}+V^{\chi +1}+E^{\chi +1}+I^{\chi +1}\right)+\mu_{1}+d+\eta_{1}+\theta +3\mu_{2}+\eta_{2}+\delta +A+\frac{b}{\tau }+M\left(\frac{\sigma_{3}^{2}}{2}+\mu_{2}+\delta +\frac{b}{\tau }\right)+M\beta I\left(c_{2}+\varepsilon +\frac{1+\varepsilon }{M}\right)+\frac{\sigma_{1}^{2}+\sigma_{2}^{2}+\sigma_{3}^{2}+\sigma_{4}^{2}}{2}\leq -\frac{1}{4}\left[\mu -\frac{1}{2}\chi \left(\sigma_{1}^{2}\vee \sigma_{2}^{2}\vee \sigma_{3}^{2}\vee \sigma_{4}^{2}\vee \sigma_{5}^{2}\right)\right]S_{1}^{\chi +1}+G\leq -\frac{1}{4}\left[\mu -\frac{1}{2}\chi \left(\sigma_{1}^{2}\vee \sigma_{2}^{2}\vee \sigma_{3}^{2}\vee \sigma_{4}^{2}\vee \sigma_{5}^{2}\right)\right]\frac{1}{\varepsilon_{1}^{\chi +1}}+G, \end{array}$$

where

(68) $$\begin{array}{c} G=\underset{\left(S_{1},S_{2},V,E,I\right)\in {\mathbb{R}}_{+}^{5}}{\sup}\left\{-\frac{1}{4}\left[\mu -\frac{1}{2}\chi \left(\sigma_{1}^{2}\vee \sigma_{2}^{2}\vee \sigma_{3}^{2}\vee \sigma_{4}^{2}\vee \sigma_{5}^{2}\right)\right]S_{1}^{\chi +1}-\frac{1}{2}\left[\mu -\frac{1}{2}\chi \left(\sigma_{1}^{2}\vee \sigma_{2}^{2}\vee \sigma_{3}^{2}\vee \sigma_{4}^{2}\vee \sigma_{5}^{2}\right)\right]\times \left(S_{2}^{\chi +1}+V^{\chi +1}+E^{\chi +1}+I^{\chi +1}\right)+\mu_{1}+d+\eta_{1}+\theta +3\mu_{2}+\eta_{2}+\delta +A+\frac{b}{\tau }+M\left(\frac{\sigma_{3}^{2}}{2}+\mu_{2}+\delta +\frac{b}{\tau }\right)+M\beta I\left(c_{2}+\varepsilon +\frac{1+\varepsilon }{M}\right)+\frac{\sigma_{1}^{2}+\sigma_{2}^{2}+\sigma_{3}^{2}+\sigma_{4}^{2}}{2}\right\}. \end{array}$$

By (53), we conclude that *LV* ≤ −1 *on* *D*_6_.

**Case 7 .**

If (*S*_1_, *S*_2_, *V*, *E*, *I*) ∈ *D*_7_, one can see that

(69) $$\begin{array}{c} LV\leq -\frac{1}{4}\left[\mu -\frac{1}{2}\chi \left(\sigma_{1}^{2}\vee \sigma_{2}^{2}\vee \sigma_{3}^{2}\vee \sigma_{4}^{2}\vee \sigma_{5}^{2}\right)\right]S_{2}^{\chi +1}-\frac{1}{4}\left[\mu -\frac{1}{2}\chi \left(\sigma_{1}^{2}\vee \sigma_{2}^{2}\vee \sigma_{3}^{2}\vee \sigma_{4}^{2}\vee \sigma_{5}^{2}\right)\right]\times S_{2}^{\chi +1}-\frac{1}{2}\left[\mu -\frac{1}{2}\chi \left(\sigma_{1}^{2}\vee \sigma_{2}^{2}\vee \sigma_{3}^{2}\vee \sigma_{4}^{2}\vee \sigma_{5}^{2}\right)\right]\left(S_{1}^{\chi +1}+V^{\chi +1}+E^{\chi +1}+I^{\chi +1}\right)+\mu_{1}+d+\eta_{1}+\theta +3\mu_{2}+\eta_{2}+\delta +A+\frac{b}{\tau }+M\left(\frac{\sigma_{3}^{2}}{2}+\mu_{2}+\delta +\frac{b}{\tau }\right)+M\beta I\left(c_{2}+\varepsilon +\frac{1+\varepsilon }{M}\right)+\frac{\sigma_{1}^{2}+\sigma_{2}^{2}+\sigma_{3}^{2}+\sigma_{4}^{2}}{2}\leq -\frac{1}{4}\left[\mu -\frac{1}{2}\chi \left(\sigma_{1}^{2}\vee \sigma_{2}^{2}\vee \sigma_{3}^{2}\vee \sigma_{4}^{2}\vee \sigma_{5}^{2}\right)\right]S_{2}^{\chi +1}+H\leq -\frac{1}{4}\left[\mu -\frac{1}{2}\chi \left(\sigma_{1}^{2}\vee \sigma_{2}^{2}\vee \sigma_{3}^{2}\vee \sigma_{4}^{2}\vee \sigma_{5}^{2}\right)\right]\frac{1}{\varepsilon_{2}^{\chi +1}}+H, \end{array}$$

where

(70) $$\begin{array}{c} H=\underset{\left(S_{1},S_{2},V,E,I\right)\in {\mathbb{R}}_{+}^{5}}{\sup}\left\{-\frac{1}{4}\left[\mu -\frac{1}{2}\chi \left(\sigma_{1}^{2}\vee \sigma_{2}^{2}\vee \sigma_{3}^{2}\vee \sigma_{4}^{2}\vee \sigma_{5}^{2}\right)\right]S_{2}^{\chi +1}-\frac{1}{2}\left[\mu -\frac{1}{2}\chi \left(\sigma_{1}^{2}\vee \sigma_{2}^{2}\vee \sigma_{3}^{2}\vee \sigma_{4}^{2}\vee \sigma_{5}^{2}\right)\right]\times \left(S_{1}^{\chi +1}+V^{\chi +1}+E^{\chi +1}+I^{\chi +1}\right)+\mu_{1}+d+\eta_{1}+\theta +3\mu_{2}+\eta_{2}+\delta +A+\frac{b}{\tau }+M\left(\frac{\sigma_{3}^{2}}{2}+\mu_{2}+\delta +\frac{b}{\tau }\right)+M\beta I\left(c_{2}+\varepsilon +\frac{1+\varepsilon }{M}\right)+\frac{\sigma_{1}^{2}+\sigma_{2}^{2}+\sigma_{3}^{2}+\sigma_{4}^{2}}{2}\right\}. \end{array}$$

Together with (54), we can deduce that *LV* ≤ −1 *on* *D*_7_.

**Case 8 .**

If (*S*_1_, *S*_2_, *V*, *E*, *I*) ∈ *D*_8_, one can see that

(71) $$\begin{array}{c} LV\leq -\frac{1}{4}\left[\mu -\frac{1}{2}\chi \left(\sigma_{1}^{2}\vee \sigma_{2}^{2}\vee \sigma_{3}^{2}\vee \sigma_{4}^{2}\vee \sigma_{5}^{2}\right)\right]E^{\chi +1}-\frac{1}{4}\left[\mu -\frac{1}{2}\chi \left(\sigma_{1}^{2}\vee \sigma_{2}^{2}\vee \sigma_{3}^{2}\vee \sigma_{4}^{2}\vee \sigma_{5}^{2}\right)\right]\times E^{\chi +1}-\frac{1}{2}\left[\mu -\frac{1}{2}\chi \left(\sigma_{1}^{2}\vee \sigma_{2}^{2}\vee \sigma_{3}^{2}\vee \sigma_{4}^{2}\vee \sigma_{5}^{2}\right)\right]\left(S_{1}^{\chi +1}+S_{2}^{\chi +1}+V^{\chi +1}+I^{\chi +1}\right)+\mu_{1}+d+\eta_{1}+\theta +3\mu_{2}+\eta_{2}+\delta +A+\frac{b}{\tau }+M\left(\frac{\sigma_{3}^{2}}{2}+\mu_{2}+\delta +\frac{b}{\tau }\right)+M\beta I\left(c_{2}+\varepsilon +\frac{1+\varepsilon }{M}\right)+\frac{\sigma_{1}^{2}+\sigma_{2}^{2}+\sigma_{3}^{2}+\sigma_{4}^{2}}{2}\leq -\frac{1}{4}\left[\mu -\frac{1}{2}\chi \left(\sigma_{1}^{2}\vee \sigma_{2}^{2}\vee \sigma_{3}^{2}\vee \sigma_{4}^{2}\vee \sigma_{5}^{2}\right)\right]E^{\chi +1}+J\leq -\frac{1}{4}\left[\mu -\frac{1}{2}\theta \left(\sigma_{1}^{2}\vee \sigma_{2}^{2}\vee \sigma_{3}^{2}\vee \sigma_{4}^{2}\vee \sigma_{5}^{2}\right)\right]\frac{1}{\varepsilon_{4}^{\chi +1}}+J, \end{array}$$

where

(72) $$\begin{array}{c} J=\underset{\left(S_{1},S_{2},V,E,I\right)\in {\mathbb{R}}_{+}^{5}}{\sup}\left\{-\frac{1}{4}\left[\mu -\frac{1}{2}\chi \left(\sigma_{1}^{2}\vee \sigma_{2}^{2}\vee \sigma_{3}^{2}\vee \sigma_{4}^{2}\vee \sigma_{5}^{2}\right)\right]E^{\chi +1}-\frac{1}{2}\left[\mu -\frac{1}{2}\chi \left(\sigma_{1}^{2}\vee \sigma_{2}^{2}\vee \sigma_{3}^{2}\vee \sigma_{4}^{2}\vee \sigma_{5}^{2}\right)\right]\times \left(S_{1}^{\chi +1}+S_{2}^{\chi +1}+V^{\chi +1}+I^{\chi +1}\right)+\mu_{1}+d+\eta_{1}+\theta +3\mu_{2}+\eta_{2}+\delta +A+\frac{b}{\tau }+M\left(\frac{\sigma_{3}^{2}}{2}+\mu_{2}+\delta +\frac{b}{\tau }\right)+M\beta I\left(c_{2}+\varepsilon +\frac{1+\varepsilon }{M}\right)+\frac{\sigma_{1}^{2}+\sigma_{2}^{2}+\sigma_{3}^{2}+\sigma_{4}^{2}}{2}\right\}. \end{array}$$

which together with (55) implies that *LV* ≤ −1 *on* *D*_8_.

**Case 9 .**

If (*S*_1_, *S*_2_, *V*, *E*, *I*) ∈ *D*_9_, we obtain

(73) $$\begin{array}{c} LV\leq -\frac{1}{4}\left[\mu -\frac{1}{2}\chi \left(\sigma_{1}^{2}\vee \sigma_{2}^{2}\vee \sigma_{3}^{2}\vee \sigma_{4}^{2}\vee \sigma_{5}^{2}\right)\right]I^{\chi +1}-\frac{1}{4}\left[\mu -\frac{1}{2}\chi \left(\sigma_{1}^{2}\vee \sigma_{2}^{2}\vee \sigma_{3}^{2}\vee \sigma_{4}^{2}\vee \sigma_{5}^{2}\right)\right]\times I^{\chi +1}-\frac{1}{2}\left[\mu -\frac{1}{2}\chi \left(\sigma_{1}^{2}\vee \sigma_{2}^{2}\vee \sigma_{3}^{2}\vee \sigma_{4}^{2}\vee \sigma_{5}^{2}\right)\right]\left(S_{1}^{\chi +1}+S_{2}^{\chi +1}+V^{\chi +1}+E^{\chi +1}\right)+\mu_{1}+d+\eta_{1}+\theta +3\mu_{2}+\eta_{2}+\delta +A+\frac{b}{\tau }+M\left(\frac{\sigma_{3}^{2}}{2}+\mu_{2}+\delta +\frac{b}{\tau }\right)+M\beta I\left(c_{2}+\varepsilon +\frac{1+\varepsilon }{M}\right)+\frac{\sigma_{1}^{2}+\sigma_{2}^{2}+\sigma_{3}^{2}+\sigma_{4}^{2}}{2}\leq -\frac{1}{4}\left[\mu -\frac{1}{2}\chi \left(\sigma_{1}^{2}\vee \sigma_{2}^{2}\vee \sigma_{3}^{2}\vee \sigma_{4}^{2}\vee \sigma_{5}^{2}\right)\right]I^{\chi +1}+K\leq -\frac{1}{4}\left[\mu -\frac{1}{2}\chi \left(\sigma_{1}^{2}\vee \sigma_{2}^{2}\vee \sigma_{3}^{2}\vee \sigma_{4}^{2}\vee \sigma_{5}^{2}\right)\right]\frac{1}{\varepsilon_{3}^{\chi +1}}+K, \end{array}$$

where

(74) $$\begin{array}{c} K=\underset{\left(S_{1},S_{2},V,E,I\right)\in {\mathbb{R}}_{+}^{5}}{\sup}\left\{-\frac{1}{4}\left[\mu -\frac{1}{2}\chi \left(\sigma_{1}^{2}\vee \sigma_{2}^{2}\vee \sigma_{3}^{2}\vee \sigma_{4}^{2}\vee \sigma_{5}^{2}\right)\right]I^{\chi +1}-\frac{1}{2}\left[\mu -\frac{1}{2}\chi \left(\sigma_{1}^{2}\vee \sigma_{2}^{2}\vee \sigma_{3}^{2}\vee \sigma_{4}^{2}\vee \sigma_{5}^{2}\right)\right]\times \left(S_{1}^{\chi +1}+S_{2}^{\chi +1}+V^{\chi +1}+E^{\chi +1}\right)+\mu_{1}+d+\eta_{1}+\theta +3\mu_{2}+\eta_{2}+\delta +A+\frac{b}{\tau }+M\left(\frac{\sigma_{3}^{2}}{2}+\mu_{2}+\delta +\frac{b}{\tau }\right)+M\beta I\left(c_{2}+\varepsilon +\frac{1+\varepsilon }{M}\right)+\frac{\sigma_{1}^{2}+\sigma_{2}^{2}+\sigma_{3}^{2}+\sigma_{4}^{2}}{2}\right\}. \end{array}$$

By (56), we can conclude that *LV* ≤ −1 on *D*_9_.

**Case 10 .**

If (*S*_1_, *S*_2_, *V*, *E*, *I*) ∈ *D*_10_, it follows that

(75) $$\begin{array}{c} LV\leq -\frac{1}{4}\left[\mu -\frac{1}{2}\chi \left(\sigma_{1}^{2}\vee \sigma_{2}^{2}\vee \sigma_{3}^{2}\vee \sigma_{4}^{2}\vee \sigma_{5}^{2}\right)\right]V^{\chi +1}-\frac{1}{4}\left[\mu -\frac{1}{2}\chi \left(\sigma_{1}^{2}\vee \sigma_{2}^{2}\vee \sigma_{3}^{2}\vee \sigma_{4}^{2}\vee \sigma_{5}^{2}\right)\right]\times V^{\chi +1}-\frac{1}{2}\left[\mu -\frac{1}{2}\chi \left(\sigma_{1}^{2}\vee \sigma_{2}^{2}\vee \sigma_{3}^{2}\vee \sigma_{4}^{2}\vee \sigma_{5}^{2}\right)\right]\left(S_{1}^{\chi +1}+S_{2}^{\chi +1}+E^{\chi +1}+I^{\chi +1}\right)+\mu_{1}+d+\eta_{1}+\theta +3\mu_{2}+\eta_{2}+\delta +A+\frac{b}{\tau }+M\left(\frac{\sigma_{3}^{2}}{2}+\mu_{2}+\delta +\frac{b}{\tau }\right)+M\beta I\left(c_{2}+\varepsilon +\frac{1+\varepsilon }{M}\right)+\frac{\sigma_{1}^{2}+\sigma_{2}^{2}+\sigma_{3}^{2}+\sigma_{4}^{2}}{2}\leq -\frac{1}{4}\left[\mu -\frac{1}{2}\chi \left(\sigma_{1}^{2}\vee \sigma_{2}^{2}\vee \sigma_{3}^{2}\vee \sigma_{4}^{2}\vee \sigma_{5}^{2}\right)\right]V^{\chi +1}+L\leq -\frac{1}{4}\left[\mu -\frac{1}{2}\chi \left(\sigma_{1}^{2}\vee \sigma_{2}^{2}\vee \sigma_{3}^{2}\vee \sigma_{4}^{2}\vee \sigma_{5}^{2}\right)\right]\frac{1}{\varepsilon_{5}^{\chi +1}}+L, \end{array}$$

where

(76) $$\begin{array}{c} L=\underset{\left(S_{1},S_{2},V,E,I\right)\in {\mathbb{R}}_{+}^{5}}{\sup}\left\{-\frac{1}{4}\left[\mu -\frac{1}{2}\chi \left(\sigma_{1}^{2}\vee \sigma_{2}^{2}\vee \sigma_{3}^{2}\vee \sigma_{4}^{2}\vee \sigma_{5}^{2}\right)\right]V^{\chi +1}-\frac{1}{2}\left[\mu -\frac{1}{2}\chi \left(\sigma_{1}^{2}\vee \sigma_{2}^{2}\vee \sigma_{3}^{2}\vee \sigma_{4}^{2}\vee \sigma_{5}^{2}\right)\right]\times \left(S_{1}^{\chi +1}+S_{2}^{\chi +1}+E^{\chi +1}+I^{\chi +1}\right)+\mu_{1}+d+\eta_{1}+\theta +3\mu_{2}+\eta_{2}+\delta +A+\frac{b}{\tau }+M\left(\frac{\sigma_{3}^{2}}{2}+\mu_{2}+\delta +\frac{b}{\tau }\right)+M\beta I\left(c_{2}+\varepsilon +\frac{1+\varepsilon }{M}\right)+\frac{\sigma_{1}^{2}+\sigma_{2}^{2}+\sigma_{3}^{2}+\sigma_{4}^{2}}{2}\right\}. \end{array}$$

Combining with (57) yields *LV* ≤ −1 on *D*_10_.

Obviously, *A*_2_ in Lemma 2.1 is satisfied. According to Lemma 2.1, we can obtain that system (4) is ergodic and has a unique stationary distribution.

**Remark 1 .**

Theorem 3 reveals that system (4) has a unique ergodic stationary distribution *π*(·) if *R*_0_^*s*^ = *η*_1_*η*_2_*βεθ*/((*μ*_1_ + *d* + *η*_1_ + (*σ*_1_^2^/2))(*θ* + *μ*_2_ + (*σ*_2_^2^/2))(*μ*_2_ + *η*_2_ + (*σ*_4_^2^/2))(*μ*_2_ + *c* + (*σ*_5_^2^/2))) > 1. Note that the expression of *R*_0_^*s*^ coincide with the threshold *R*_0_ of the deterministic system (1) if there is no stochastic perturbation. This shows that we generalize the result of the deterministic system.

### 3.3. Extinction of the Disease

As it is well known, one of the main concern of epidemiology is how we regulate the disease dynamics in order to eradicate the disease in the long term. Moreover, in [10], Allen et al. proposed and studied several types of stochastic epidemic models and pointed out that the stochastic models should suit the question of disease extinction better. Hence, in this section, we shall establish some sufficient conditions for extinction of the disease in stochastic model (4).

**Theorem 3 .**

Let *S*_1_(*t*), *S*_2_(*t*), *V*(*t*), *E*(*t*), *I*(*t*) be the solution of system (4) with any initial value (*S*_1_(0), *S*_2_(0), *V*(0), *E*(0), *I*(0)) ∈ ℝ_+_^5^. If (*β*(*ε* + 1)(*Aτ* + *b*)(*μ*_2_ + *η*_2_))/*μτη*_2_ < ((*σ*_5_^2^/2) + *μ*_2_ + *c*)∧(*σ*_4_^2^/2), then the disease *I*(*t*) will extinct exponentially with probability one, i.e., moreover

(77) $$\begin{array}{c} \underset{t⟶\infty }{\lim}\sup\frac{1}{t}\log\left[E+\frac{\mu_{2}+\eta_{2}}{\eta_{2}}I\right]\leq \frac{\beta \eta_{2}\left(\varepsilon +1\right)\left(A\tau +b\right)}{\left(\mu_{2}+\eta_{2}\right)\mu \tau }-{\left(\frac{\eta_{2}}{\mu_{2}+\eta_{2}}\right)}^{2}\left[\left(\frac{\sigma_{5}^{2}}{2}+\mu_{2}+c\right)\wedge \left(\frac{\sigma_{4}^{2}}{2}\right)\right]. \end{array}$$

**Proof**

Applying It$\hat{o}$'s formula to log[*E* + (*μ*_2_ + *η*_2_/*η*_2_)*I*], we have

(78) $$\begin{array}{c} d\log\left[E+\frac{\mu_{2}+\eta_{2}}{\eta_{2}}I\right]=\left[\frac{\beta \left(\varepsilon V+S_{2}\right)I}{E+\left(\mu_{2}+\eta_{2}/\eta_{2}\right)I}-\frac{\left(\mu_{2}+\eta_{2}\right)\left(\mu_{2}+c\right)I}{\left(E+\left(\mu_{2}+\eta_{2}/\eta_{2}\right)I\right)\eta_{2}}-\frac{\sigma_{4}^{2}E^{2}+\sigma_{5}^{2}\left(\left(\mu_{2}+\eta_{2}/\eta_{2}\right)\right)I^{2}}{2{\left(E+\left(\mu_{2}+\eta_{2}/\eta_{2}\right)I\right)}^{2}}\right]dt+\frac{\sigma_{4}E}{E+\left(\mu_{2}+\eta_{2}/\eta_{2}\right)I}dB_{4}\left(t\right)+\frac{\sigma_{5}\left(\mu_{2}+\eta_{2}\right)I}{\eta_{2}\left(E+\left(\mu_{2}+\eta_{2}/\eta_{2}\right)I\right)}dB_{5}\left(t\right)=\frac{\beta \left(\varepsilon V+S_{2}\right)I}{E+\left(\mu_{2}+\eta_{2}/\eta_{2}\right)I}dt-\frac{1}{{\left(E+\left(\mu_{2}+\eta_{2}/\eta_{2}\right)I\right)}^{2}}\left[\left(\frac{\mu_{2}+\eta_{2}}{\eta_{2}}\right)\left(\mu_{2}+c\right)IE+\left(\frac{\sigma_{5}^{2}}{2}+\mu_{2}+c\right){\left(\frac{\mu_{2}+\eta_{2}}{\eta_{2}}\right)}^{2}I^{2}+\frac{\sigma_{4}^{2}E^{2}}{2}\right]dt+\frac{\sigma_{4}E}{E+\left(\mu_{2}+\eta_{2}/\eta_{2}\right)I}dB_{4}\left(t\right)+\frac{\sigma_{5}\left(\mu_{2}+\eta_{2}\right)I}{\eta_{2}\left(E+\left(\mu_{2}+\eta_{2}/\eta_{2}\right)I\right)}dB_{5}\left(t\right)\leq \frac{\beta \left(\varepsilon V+S_{2}\right)\eta_{2}}{\mu_{2}+\eta_{2}}dt-\frac{1}{{\left(E+\left(\mu_{2}+\eta_{2}/\eta_{2}\right)I\right)}^{2}}\left[\left(\frac{\sigma_{5}^{2}}{2}+\mu_{2}+c\right){\left(\frac{\mu_{2}+\eta_{2}}{\eta_{2}}\right)}^{2}I^{2}+\frac{\sigma_{4}^{2}E^{2}}{2}\right]dt+\frac{\sigma_{4}E}{E+\left(\mu_{2}+\eta_{2}/\eta_{2}\right)I}dB_{4}\left(t\right)+\frac{\sigma_{5}\left(\mu_{2}+\eta_{2}\right)I}{\eta_{2}\left(E+\left(\mu_{2}+\eta_{2}/\eta_{2}\right)I\right)}dB_{5}\left(t\right)\leq \frac{\beta \eta_{2}\left(\varepsilon +1\right)\left(A\tau +b\right)}{\left(\mu_{2}+\eta_{2}\right)A\tau }dt-{\left(\frac{\eta_{2}}{\mu_{2}+\eta_{2}}\right)}^{2}\left[\left(\frac{\sigma_{5}^{2}}{2}+\mu_{2}+c\right)\wedge \left(\frac{\sigma_{4}^{2}}{2}\right)\right]dt+\frac{\sigma_{4}E}{E+\left(\mu_{2}+\eta_{2}/\eta_{2}\right)I}dB_{4}\left(t\right)+\frac{\sigma_{5}\left(\mu_{2}+\eta_{2}\right)I}{\eta_{2}\left(E+\left(\mu_{2}+\eta_{2}/\eta_{2}\right)I\right)}dB_{5}\left(t\right). \end{array}$$

Integrating the above inequality from 0 to *t*, and the fact that lim_*t*⟶∞_*B*_*i*_(*t*)/*t* = 0, *i* = 4, 5 [16], yields

(79) $$\begin{array}{c} \lim_{t⟶\infty }\sup\frac{1}{t}\log\left[E+\frac{\mu_{2}+\eta_{2}}{\eta_{2}}I\right]\leq \frac{\beta \eta_{2}\left(\varepsilon +1\right)\left(A\tau +b\right)}{\left(\mu_{2}+\eta_{2}\right)\mu \tau }-{\left(\frac{\eta_{2}}{\mu_{2}+\eta_{2}}\right)}^{2}\left[\left(\frac{\sigma_{5}^{2}}{2}+\mu_{2}+c\right)\wedge \left(\frac{\sigma_{4}^{2}}{2}\right)\right]=x_{0}. \end{array}$$

For any $\bar{\varepsilon }>0$, and almost *ω* ∈ *Ω*, ∃*T* = *T*(*ω*) such that

(80) $$\begin{array}{c} I\left(t\right)\leq \frac{\eta_{2}}{\mu_{2}+\eta 2}\exp\left(\left(x_{0}+\bar{\varepsilon }\right)t\right),\forall t\geq T. \end{array}$$

**Remark 2 .**

Theorem 5 suggests that the disease will become extinct if (*β*(*ε* + 1)(*Aτ* + *b*)(*μ*_2_ + *η*_2_))/*μτη*_2_ < ((*σ*_5_^2^/2) + *μ*_2_ + *c*)∧(*σ*_4_^2^/2).

## 4. Numerical Examples

In this section, we will give two numerical examples to illustrate the main theoretical results obtained in this paper. The numerical simulation method can be found in [9, 22, 23]. The following is a corresponding discrete equations of system (4):

(81) $$\begin{array}{c} \begin{array}{c} S_{1k+1}=S_{1k}+\left[A+\frac{b\left(S_{2k}+V_{k}\right)}{1+\tau \left(S_{2k}+V_{k}\right)}-\left(\mu_{1}+d+\eta_{1}\right)S_{1k}\right]\Delta t+S_{1k}\left[\sigma_{1}\xi_{k}\sqrt{\Delta t}+\frac{1}{2}\sigma_{1}^{2}\left(\xi_{k}^{2}-1\right)\Delta t\right],\\ S_{2k+1}=S_{2k}+\left[\eta_{1}S_{1k}-\beta S_{2k}I_{k}-\theta S_{2k}-\mu_{2}S_{2k}+\delta V_{k}\right]\Delta t+S_{2k}\left[\sigma_{2}\xi_{k}\sqrt{\Delta t}+\frac{1}{2}\sigma_{2}^{2}\left(\xi_{k}^{2}-1\right)\Delta t\right],\\ V_{k+1}=V_{k}+\left[\theta S_{2k}-\varepsilon \beta V_{k}I_{k}-\left(\mu_{2}+\delta \right)V_{k}\right]\Delta t+V_{k}\left[\sigma_{3}\xi_{k}\sqrt{\Delta t}+\frac{1}{2}\sigma_{3}^{2}\left(\xi_{k}^{2}-1\right)\Delta t\right],\\ E_{k+1}=E_{k}+\left[\beta \varepsilon V_{k}I_{k}+\beta S_{2k}I_{k}-\left(\mu_{2}+\eta_{2}\right)E_{k}\right]\Delta t+E_{k}\left[\sigma_{4}\xi_{k}\sqrt{\Delta t}+\frac{1}{2}\sigma_{4}^{2}\left(\xi_{k}^{2}-1\right)\Delta t\right],\\ I_{k+1}=I_{k}+\left[\eta_{2}E_{k}-\left(\mu_{2}+c\right)I_{k}\right]\Delta t+I_{k}\left[\sigma_{5}\xi_{k}\sqrt{\Delta t}+\frac{1}{2}\sigma_{5}^{2}\left(\xi_{k}^{2}-1\right)\Delta t\right], \end{array} \end{array}$$

where *ξ*_*k*_ (*k* = 1, 2, ⋯) are the Gaussian random variables which follow standard normal distribution *N*(0, 1), and *σ*_*i*_, 1 ≤ *i* ≤ 5, are intensities of white noises.

**Example 1 .**

We take parameters as *A* = 45, *β* = 0.05, *μ*_1_ = 0.05, *μ*_2_ = 0.06, *ε* = 3.2, *τ* = 0.01, *b* = 0.3, *η*_1_ = 0.25, *η*_2_ = 0.5, and *θ* = 1.1, *δ* = 0.01, *c* = 0.02, *σ*_1_ = 0.2, *σ*_2_ = 0.05, *σ*_3_ = 0.31, *σ*_4_ = 0.03, and *σ*_5_ = 0.02. It is clear that conditions of Theorem 3 are satisfied; by calculating, we have the basic reproduction number *R*_0_^*s*^ = *η*_1_*η*_2_*βεθ*/((*μ*_1_ + *d* + *η*_1_ + (*σ*_1_^2^/2))(*θ* + *μ*_2_ + (*σ*_2_^2^/2))(*μ*_2_ + *η*_2_ + (*σ*_4_^2^/2))(*μ*_2_ + *c* + (*σ*_5_^2^/2))) = 1.17080128

The histogram and the smoothing curves of the probability density functions of *S*_1_(*t*), *S*_2_(*t*), *V*(*t*), *E*(*t*), *I*(*t*) are given in Figure 1.

**Example 2 .**

We take parameters as *A* = 1000, *β* = 0.0001, *μ*_1_ = 0.1, *μ*_2_ = 0.25*ε* = 0.18, *τ* = 0.002, *b* = 1.5, *η*_1_ = 1.06, *η*_2_ = 3.4, and *θ* = 0.1, *δ* = 0.4, *c* = 0.05, *σ*_1_ = 0.2, *σ*_2_ = 0.5, *σ*_3_ = 0.31, *σ*_4_ = 1.65, and *σ*_5_ = 1.5. It is clear that conditions of Theorem 5 are satisfied.

The curves on the persistence of *S*_1_(*t*), *S*_2_(*t*), *V*(*t*), *E*(*t*) and extinction of *I*(*t*) for stochastic model (4) are given in Figure 2, where the initial value is (*S*_1_(0), *S*_2_(0), *V*(0), *E*(0), *I*(0)) = (1,1.5,1, 1, 1).

**Remark 3 .**

In this paper, we consider the stochastic perturbations for deterministic model (1) and derived model (4). Thus, model (4) can be specialized as models (1). Hence, model (4) can be seen as a general model compared to model (1), and the theoretical results obtained in this article can be seen as the extensions and supplements of the model and the theoretical results obtained in [8].

## 5. Conclusion

In this paper, firstly, we have considered the stochastic perturbations for deterministic system (1) and established corresponding stochastic system (4). Secondly, under the condition *R*_0_^*s*^ > 1 and applying the theory of stochastic differential equations, Has'minskii theory, Ito's formula, and Lyapunov function method, we obtained some sufficient conditions on the existence of ergodic stationary distribution of model (4). We also established sufficient conditions on the extinction of the disease. Finally, two examples are presented to validate the main results of this paper. The results obtained in this paper suggest that stochastic perturbations have remarkable effects on the disease in model (4). Especially, from the numerical simulations, we can see that, under the stochastic perturbations, the disease in the stochastic system will become extinct more quickly than the corresponding deterministic one.

## Figures and Tables

**Figure 1:** Dynamic behaviors of the system.

**Figure 2:** Dynamic behaviors of the system.

## Data Availability

No data were used to support this study.
